# A Research on the Realization Algorithm of Internet of Things Function for Smart Education

This article has been retracted.

**DOI:** 10.1155/2022/1330190

**Published:** 2022-04-29

**Authors:** Kuiliang Fu

**Affiliations:** College of Health Engineering, Nanjing City Vocational College, Nanjing 211200, China

## Abstract

The traditional teaching mode is to use a point-to-point mode or a computer-aided system for teaching, but this limits students' enthusiasm and interest in learning. The Internet of Things (IoT) technology is a technology that integrates sensors, the Internet, and terminals to transmit information in real time. The smart education based on the Internet of Things can realize remote teaching and actual scene teaching, and students can freely choose the learning location and time, which can greatly improve students learning interest and learning efficiency, which is a development trend of a new teaching method. Smart IoT teaching is a teaching method that combines IoT technology and artificial intelligence technology. This paper mainly studies the research and analysis of the smart education model based on the IoT in remote teaching. In this paper, sensor technologies such as cameras will be used to collect students' expressions, speech, and other actions in class from different regions. These data features will be processed by the terminal's intelligent algorithm, and the desired knowledge will be obtained according to the students' behavior information. The information processed by the intelligent algorithm will be transmitted to the terminal system where the teacher is located, such as computer and mobile phone. This paper focuses on analyzing the reliability and accuracy of the intelligent algorithm of the IoT smart education terminal. The results show that the prediction error of the student behavior information is within 3% and the correlation coefficient reaches 0.99.

## 1. Introduction

The traditional teaching mode is often a point-to-point teaching mode, in which teachers transmit knowledge to students in one way through textbooks. In recent years, the development of computer-aided systems has also promoted the change of teaching mode [1]. It can display knowledge to students more intuitively, which stimulates students' interest in learning and understanding. However, neither of these two teaching modes can generate real-time interaction, and it is also difficult to generate new teaching content in time according to students' learning interests. They also limit the use of students' imaginations, which in turn limits the extent to which knowledge can be expanded [2, 3]. At the same time, there is a problem of uneven distribution of education in China, which makes it difficult for students in underdeveloped areas to receive advanced knowledge. If the classroom can realize remote education through the Internet of Things technology, it will not only save teachers' time cost, and students can interact with teachers in different places for the first time [4]. With the rapid development of the Internet of Things and artificial intelligence, this kind of Internet-based smart remote education is relatively easy to implement [5]. It can solve some defects of the traditional education model and the computer-aided system education model, and at the same time, it will greatly improve students' learning fun and range of knowledge.

The Internet of Things technology is the product of the third scientific and technological revolution of information technology [6]. It connects the controlled objects, sensor equipment, cloud computing, Internet terminals, and other types of equipment according to certain protocols and then realizes remote intelligent identification on mobile phones or computer terminals [7], control, positioning, supervision, and other functions of technology. The Internet of Things technology is also a product that can be compared with artificial intelligence technology. It has been widely used in transportation, agriculture, medicine, and other fields. In the field of education, the application of IoT technology is relatively small, mostly in the research stage. If the Internet of Things technology and artificial intelligence technology are combined, the wisdom of education will be realized, which is called wisdom education [8]. This method can realize the real-time push of appropriate knowledge according to students' behavior information in the process of remote teaching [9], which can increase the richness of the classroom and improve students' desire for knowledge. The rapid development of artificial intelligence technology and the continuous improvement of hardware equipment such as sensors provide reliable technical support for the development and application of smart education [10]. This research mainly uses the neural network method combined with the Internet of Things technology to realize the smart teaching method in remote teaching.

The education model has gone through the stages of point-to-point teaching, computer-aided system teaching, and so on. In recent years, many studies have been carried out on education methods based on artificial intelligence methods or Internet of Things technology. Zhang et al. [11] believed that smart education is interactive knowledge and a generalized higher education model. Based on the AIISE, an artificial intelligence-assisted interactive intelligent education framework, they changed students' enthusiasm for classroom interaction, and it can be concluded that the artificial intelligence-assisted student interactive teaching model improved students' performance. Majeed and Ali [12] designed a smart teaching system on a university campus based on the Internet of Things system, which is mainly composed of sensors, controllers, physical objects, and so on. The communication between them is completed by the Internet. Various sensors are connected to physical objects, and wearable technology is used to enhance the collected datasets. Their research results show that this smart education model improves the interactivity of college students' classrooms. Han and Xu [13] believed that smart teaching should be integrated into the learning environment and educational environment, and it can demonstrate an innovative application and new teaching ideas. Based on the powerful image recognition and detection function of deep learning DL, they designed an automatic intelligent teaching method that integrates teaching evaluation and teaching design. They proposed a smart teaching system based on ecological evaluation, a platform that can perceive students' perceptions in real time for educational evaluation and development. Mohammadian et al. [14] believed that the integration of the Internet of Things and education is a disruptive innovative technology that will fundamentally solve the way of education management, interaction, and control. They designed a new type of IoT intelligent teaching method in response to the needs of the German IoT intelligent development SME4.0 environment. At the same time, they proposed the implementation method of educational infrastructure according to the Internet of Things technology. Chen et al. [15] proposed a multisensor information fusion technology based on the Kalman filter technology, which integrates IoT technology and sensors. At the same time, they designed and integrated the system with wireless network technology. They combined the new information sensor fusion technology with the Internet of Things to design a smart education system and carried out experimental verification steps. The conclusion shows that this system has certain feasibility, and it can improve the efficiency of smart classroom. Kusmin and Laanpere [16] integrated IoT technology into the learning process of education. At the same time, they combined inquiry-based learning (IBL) and problem-based learning (PBL) with IoT devices (sensors, terminals, Internet, etc.) and interdisciplinary education to design a new IoT smart education system. This system is also used as an actual instructional design experiment. It can reflect relevant knowledge and suggestions to teachers according to the problems encountered by students in the learning process. In response to the problems of slow response and poor teaching efficiency of related platforms in the English teaching classroom, Liu and Yang [17] proposed an innovative English teaching platform based on the Internet. This platform will integrate the student cloud platform, the teacher cloud platform, the interactive classroom platform, and so on. It uses the fuzzy hierarchical evaluation model to evaluate the actual test of the system. The results show that the delay of this IoT smart English teaching platform is less than 0.3 s and the overall satisfaction is 9.2 points. Liu et al. [18] designed a smart education system based on the Internet of Things technology and traditional network, which can realize functions such as online score query, online teaching, and teaching management. This system has a hierarchical structure layer. The experimental results show that this IoT smart education platform has the advantages of high throughput and low latency. Others have also conducted a lot of research on the integration of the Internet of Things and smart education, but these studies mainly use the Internet of Things and innovative sensor technologies or new application levels to integrate [19–23], and few smart education systems involve artificial intelligence technology with the Internet of Things. Through the above review, it can be found that the current research has begun to conduct a lot of research on smart education, which will promote the development of education and the improvement of learning efficiency. However, the current research has not really realized the organic integration of the Internet of Things and smart education. This paper proposes a smart education model that combines the Internet of Things and artificial intelligence to address the shortcomings of educational methods.

From the above literature, it can be seen that the current research on smart education mainly adopts artificial intelligence methods or Internet of Things technology to realize smart education systems, such as the image detection function of deep learning or the role of sensors and cloud computing of Internet of Things technology [24–26]. However, most of the studies do not really consider the behavioral information of students in the classroom and then propose the learning content of interest [27]. This research is mainly based on the multisensor fusion Internet of Things technology and artificial intelligence technology to realize the smart teaching system. The main research object is remote smart education in remote teaching. First, audio-visual sensors are used to collect classroom behavior information of students in multiple regions. This information will be transmitted to the teaching terminal through the Internet, and the terminal will use the deep learning intelligent algorithm to process and output the data.

The research on the integration of the Internet of Things and smart teaching methods will be introduced in five parts. The first part mainly introduces the development status of the Internet of Things and the development status of smart education. The second part mainly introduces the necessity of the integration of IoT and smart education and the data processing scheme. The third part mainly introduces the design of the IoT smart education system and the required algorithms. The fourth part is to study the accuracy of the realization of smart education algorithm. The fifth part is the summary of the paper, which mainly analyzes the current shortcomings of smart education and the advantages and accuracy of the IoT smart model proposed in this paper.

## 2. The Significance of the Integration of IoT Technology and Smart Education and the Source of Sensor Data

### 2.1. The Necessity of the Integration of IoT Technology and Smart Education

The traditional education method and the education method of the computer-aided system will limit the scope of knowledge received by students and their interest in learning knowledge [28]. At the same time, the uneven geographical distribution of education will also cause waste of educational resources. The Internet of Things technology is a way to interconnect terminals, sensors, and the Internet. It has been widely used in transportation, agriculture, medicine, and other fields and has achieved relatively efficient results [29, 30]. At the same time, in recent years, the integration of IoT technology and education has also demonstrated many researches and applications, such as applications in the form of distance classes and online education, but it is still difficult to realize the intelligence of education in this way [31]. Deep learning methods have shown good performance in the fields of image recognition and speech recognition. In remote education, there is a close connection between students' behavioral information, verbal information, and learning content in the classroom. The feature predicts the course content of interest in learning, which will not only improve students' interest in learning but also greatly improve learning efficiency, which also reduces the burden of lesson preparation for teachers [32]. This research makes full use of the advantages of distance education of the Internet of Things and the ability of deep learning to mine information features to design a smart education system of the Internet of Things.

### 2.2. The Data Sources for IoT Multisensor Systems

This research will collect classroom behavior information and speech information of students in multiple regions through the multisensor technology of the Internet of Things system as the data source for data mining of intelligent terminals. Students' interest in knowledge and their ability to accept knowledge can be reflected through classroom behaviors, which mainly include students' expressions, actions, and speech. There is a strong correlation between these actions and the teaching content. If the deep learning algorithm can extract the behavioral characteristics of students and then establish the mapping relationship with the teaching content, it will greatly improve the students' learning interest and learning efficiency. The problem of unbalanced geographical educational resources is mainly due to the close relationship between teachers' teaching methods, and the students' behavior information is also closely related to teachers' teaching methods. This can also suggest a special relationship through the nonlinear mapping capabilities of deep learning. Therefore, the sensor of the student terminal will collect the students' speech and behavior characteristics as the input data of the smart education algorithm, and the sensor of the teacher terminal will collect the teacher's behavior information and teaching content as the output of the intelligent education algorithm. A nonlinear mapping relationship is established between input and output. Ultimately, this intelligent algorithm will realize a smart teaching system for remote teaching under the combination of Internet of Things technology and deep learning technology. These data sources are collected by the sensors of the Internet of Things, which are processed by the intelligent algorithms of the terminal system of the IoT. In this paper, the student behavior information and teacher behavior information extracted by the Internet of Things multisensor system are used as the dataset, and the dataset will be divided into training set, test set, and verification set. The dataset selected in this paper is mainly derived from the multisensor system of the Internet of Things technology, which mainly includes student behavior information, speech information from the student terminal, teacher behavior information from the teacher terminal, and courseware content.

## 3. The Composition of the IoT Smart Education System and the Introduction of Smart Algorithms

### 3.1. The Composition of IoT Smart Education System

The IoT smart education system is mainly composed of IoT hardware devices and intelligent algorithms. The main purpose of the Internet of Things hardware equipment is to realize the functions of information collection, transmission, and output of students in remote classrooms. The purpose of intelligent algorithms is mainly to extract features and map correlations for the information collected by IoT hardware devices. The sensors of the IoT system mainly include cameras and recording devices. The purpose of the cameras is to collect the behavior information of students and teachers and the content of courseware. The main purpose of the recording devices is to collect the speech information of students and teachers. The transmission technology adopted by the Internet of Things technology in this paper will be transmitted in the form of a wireless network. The terminal system may take the form of a cell phone or a computer system.  Figure 1 shows the hardware device composition and information transfer process of the IoT smart education system. It can be seen that this is an information transfer system with a feedback mechanism. There is a feedback information system between student behavior information, teacher behavior information, and courseware content, which can ensure the information collection of the intelligent education system and the timely acquisition of data by the intelligent algorithm, and then the prediction function of the classroom can be performed. The working end of the Internet of Things technology mainly collects student behavior information by the camera system and audio-visual technology, then these data are transmitted to the teacher's terminal system through the Internet, and then intelligent decision-making processing is carried out on it. The intelligent decision-making algorithm of smart education will complete the training and prediction of the model on the TensorFlow platform of the computer-aided system, and the optimized weights and parameters will be saved in the computer-aided system for use in the teacher's terminal classroom.

### 3.2. IoT Multisensor Data Fusion Algorithm

The Internet of Things technology used in this study will use multiple cameras and multiple recording devices to collect data from students' classroom information in different places. These data need to be sent to the computer-aided system of the teacher's terminal through data fusion. Data fusion is the need to organize these information data features and transmit them through Internet technology with a unified feature. Data fusion technology refers to the information processing technology that uses the computer system to automatically analyze and synthesize the chronologically acquired image or audio data within certain criteria to complete decision-making and evaluation tasks. The Internet of Things technology will collect image and auditory data through a multisensor system, and these data will be fused into the computer processing system of the Internet of Things terminal so as to be transmitted to the teacher terminal auxiliary system through the Internet.

There are many ways of data fusion algorithm, such as Kalman filter or DS theory. In this paper, DS theory is used to perform data fusion on the multisensor information data of the Internet of Things. Data fusion technology is a process of collecting, transmitting, and synthesizing useful information from various information sources to assist people in planning, verifying, and determining information. This data-fused student behavior information will be input into an intelligent decision-making system.  Figure 2 shows the workflow of data fusion of IoT multisensor data source information.

DS theory is a complete theory for dealing with uncertainty. In this paper, DS theory will be used to perform data fusion on IoT multisensor data sources. It will give the comprehensive probability of each hypothesis according to the occurrence probability of different data sources and then perform data fusion on the data sources of different sensors. Equation (1) illustrates the basic theoretical probability function mass function used in the DS theory process. *A* represents the behavior information, speech information, or facial expression information of the student terminal collected by the sensor. *m* represents the probability of finding these datasets.

(1) $$\begin{array}{c} \sum_{A\subseteq \Theta }m\left(A\right)=1. \end{array}$$

The sum of the probabilities for all subsets of IoT assumptions about sensor data sources is called the belief function, and equation (2) shows the calculation rules for the belief function.

(2) $$\begin{array}{c} Bel\left(A\right)=\sum_{B\subseteq A}m\left(b\right). \end{array}$$

The sum of the probabilities that the intersection of various hypotheses about IoT multisensor data sources is not an empty set is called the likelihood function, and equation (3) shows the calculation method of the likelihood function.

(3) $$\begin{array}{c} Pl\left(A\right)=\sum_{B\cap A\neq \Phi }m\left(B\right). \end{array}$$

DS theory is also known as evidence synthesis method, and equation (4) shows the DS synthesis rule for data fusion of IoT collected data.

(4) $$\begin{array}{c} m_{1}⊕m_{2}=\frac{1}{K}\sum_{B\cap C=A}m_{1}\left(B\right)\cdot m_{2}\left(C\right). \end{array}$$

Equation (5) shows the calculation rule of *K*; that is, the sum of the products of the two assumptions after the mass function operation is divided by the normalization coefficient *K*.

(5) $$\begin{array}{c} K=1-\sum_{B\cap C\neq \Phi }m_{1}\left(B\right)\cdot m_{2}\left(C\right). \end{array}$$

The other way is to set 1 − *K* as the normalization processing coefficient, which is different from the definition of equation (5), but they contain the same meaning. Equation (6) illustrates the calculation rules of the 1 − *K* algorithm.

(6) $$\begin{array}{c} 1-K=\sum_{B\cap C\neq \Phi }m_{1}\left(B\right)\cdot m_{2}\left(C\right). \end{array}$$

### 3.3. The Introduction of Intelligent Decision Algorithms of Smart Education

The Internet of Things technology transmits student behavior information to the teacher's terminal through sensor technology and the transmission function of the Internet, which requires intelligent decision-making algorithms to predict and process this data information. In this paper, the convolutional neural network technology is used to preprocess and predict the information collected by the Internet of Things. Neural network technology has obvious advantages in processing nonlinear and high-dimensional data. Convolutional neural network can extract features of student behavior information through weight sharing and other methods and then complete nonlinear mapping through activation functions, which is very suitable for intelligent education. The information collected by both cameras and recording equipment has complex characteristics. It is difficult to map the relationship between student behavior information and students' interested knowledge by thinking. Convolutional neural networks and recurrent neural networks can be very good. To deal with the spatial correlation as well as the temporal correlation of student behavior characteristics, Figure 3 shows the workflow of the intelligent decision-making algorithm of IoT terminal devices. The student behavior information and the teacher behavior information come from the sensors of the student terminal and the teacher terminal, respectively, and they have been processed by the data fusion algorithm. These data features will be used as the input of the convolutional neural network for feature extraction.

The learning rate of 0.0001 and the number of filters of 128 were adopted by the intelligent decision-making algorithm in this study. Meanwhile, the number of layers of the neural network is set to 4. Neural network technology often finds optimal weights and biases through gradient descent methods and then optimizes research problems. These weights and biases are matrixed through a nonlinear activation function, and the predicted and actual values are backpropagated through a loss function. Equation (7) shows the basic operating rules of the neural network method.

(7) $$\begin{array}{c} x_{j}=f\left(\sum_{i\in M_{j}}x_{i}^{\zeta -1}*k_{ij}^{\zeta }+b_{j}^{\zeta }\right). \end{array}$$

The convolutional neural network method is different from the fully connected neural network method because the weights are shared, and the features do not all need to perform matrix operations with each weight, which involves the process of upsampling and downsampling. Equations (8) and (9) show the workflow of upsampling and downsampling of the pooling layer of a convolutional neural network, respectively.

(8) $$\begin{array}{c} \delta_{j}^{\zeta }=\beta_{j}^{\zeta +1}\left(f^{\prime }{\left(u\right)}_{l}^{\zeta }\circ up\left(\delta_{j}^{\zeta +1}\right)\right), \end{array}$$

(9) $$\begin{array}{c} x_{j}=f\left(\sum_{u,v}\beta_{j}^{\zeta }do\;wn\left(x_{i}^{\zeta -1}\right)+b_{j}^{\zeta }\right). \end{array}$$

The process of matrix operations and backpropagation of biases and weights involves many differential derivation operations, which are the most basic operations of neural networks. Equation (10) shows the rules of differential derivation operations. *W* is the weights, and *b* is the dataset matrix. *u* and *v* are the different dataset features.

(10) $$\begin{array}{c} \frac{\partial W}{\partial b_{j}}=\sum_{u,v}\delta_{j}^{\zeta }uv. \end{array}$$

The feature extraction of students' speech information in this study uses a recurrent neural network, which requires partial memory of historical state information. Equations (11) and (12) show the memory flow of historical state information. The input of a recurrent neural network is the temporal feature output of a convolutional neural network, which is a continuous prediction process. Recurrent neural network is mainly used to extract the temporal features of student behavior information.

(11) $$\begin{array}{c} o_{t}=\sigma \left(W_{xo}{}^{*}x_{t}+W_{ho}{}^{*}h_{t-1}+W_{co}\circ C_{t}+b_{o}\right), \end{array}$$

(12) $$\begin{array}{c} h_{t}=o_{t}\circ ELU\left(C_{t}\right). \end{array}$$

### 3.4. The Process of Collecting Data from the Internet of Things

This paper uses cameras and recording equipment to collect information from students' classrooms. It can be found that the data collected by the Internet of Things technology cannot be used by the intelligent decision-making algorithm of intelligent education, which requires preprocessing of the information collected by the Internet of Things technology. The information collected by the Internet of Things technology includes images and auditory information. Both the dimensional form of the data and the distribution of the data are inconsistent, which is unfavorable for the optimization in the intelligent decision-making stage. First, this study matrixed the images collected by IoT sensors and processed these data into data that conformed to a normal distribution and were within an interval. Then, the auditory information is also matrixed to make it consistent with the distribution and interval of the image information. This research will use the TensorFlow platform and the Keras pattern library for model training, and the weights and biases after training will be saved in h5 format.

## 4. The Feasibility Analysis and Accuracy Analysis of IoT Smart Education

The IoT smart education system is mainly composed of IoT hardware devices and intelligent decision-making parts. IoT hardware devices are mainly used to complete information adoption and interface display of terminal devices. The combination of artificial intelligence and Internet of Things technology is the key to the realization of smart education. This paper mainly analyzes the accuracy and feasibility of intelligent algorithms in the decision-making stage of smart education.  Figure 4 shows the classification proportion of educational classroom data collected by Internet of Things information collection equipment. It can be clearly seen from the figure that the proportion of student behavior information collected by Internet of Things collection equipment is relatively uniform, which is conducive to intelligent algorithms to find the optimal solution. Although there are certain differences between the four different types of student behavior information, the overall difference is relatively small, the largest proportion is 29.2%, and the smallest proportion of behavior information classification also reaches 21.2%, which is a reasonable value range. The largest proportion of student behavior information is student speech information that is more relevant to students, the smallest is mainly student behavior and action information, and other pieces of information include courseware content.  Figure 5 shows the difference between the student behavior information collected by the Internet of Things and the average value and the difference between the behavior information and the minimum value, which can reflect the distribution characteristics of the data information collected by the Internet of Things. It can be seen from Figure 5 that the difference between the student's action behavior information and speech behavior information and the mean value is relatively small, and they are distributed on both sides of the mean value, which shows that the two kinds of student behavior information collected by the Internet of Things system are evenly distributed. At the same time, the difference between the two kinds of student behavior information collected by the IoT system and the minimum value is relatively small. From the above two analyses, the student behavior information collected by the IoT system can be better input into the intelligent algorithm.

According to the process of the IoT intelligent education system designed in this paper, it can be known that the student behavior information collected by the IoT will be input into the intelligent decision-making algorithm system.  Figure 6 shows the prediction error of the intelligent decision-making algorithm of the intelligent education system. This paper selects four kinds of behavioral information, including student expressions, student speech, teacher behavior information, and courseware content, as predictions. It can be clearly seen from Figure 6 that the prediction errors of the four types of student and teacher behavior information are relatively small, which is an acceptable error range for the IoT intelligent education system. It can be seen from Figure 6 that the largest error is only 2.91%, and the smallest error is only 0.91%. The largest prediction error comes from the students' verbal information, which is mainly because the students' verbal information has obvious time characteristics and the students' verbal information is variable, which is difficult for intelligent algorithms.  Figure 7 shows the distribution of the predicted value and the actual value of the student behavior information by the intelligent algorithm of the intelligent education system in the form of polar coordinates. It can also be seen intuitively from Figure 7 that the distribution of the predicted value of the student and teacher information is relatively consistent with the actual value, and only a small part has a certain difference. From the description of Figures 6 and 7, it can be found that the intelligent algorithm adopted in this paper is more suitable for predicting the behavior information of students and teachers in the Internet of Things education system.

In this study, the box distribution map and the columnar prediction distribution map were selected as the analysis of statistical parameters.  Figure 8 shows the distribution box diagram of the predicted value and the actual value of the intelligent education decision-making algorithm. It can be seen from Figure 8 that the box size and shape of the predicted value are consistent with the box distribution of the actual value. From the distribution of the median line and the mean line in Figure 8, it can be seen that the difference between the predicted mean value of the student behavior information and the median line and the two parameter quantities of the actual student behavior information are relatively small. This can reflect that the predicted value of the intelligent decision-making algorithm has a great similarity with the actual value, whether it is the data value or the distribution shape of the data. From the columnar prediction distribution in Figure 9, it can be more clearly seen that the distribution and value of the predicted value of the student behavior information are similar to the actual value, which shows that the intelligent algorithm of the IoT intelligent education system is reliable. It can be clearly seen from Figure 9 that there is an obvious correlation between the predicted value generated by the intelligent decision-making algorithm and the data of the actual teaching mode, and the correlation coefficient basically exceeds 0.99.

## 5. Research Summary

The Internet of Things technology is a way to interconnect application objects through technologies such as multisensor systems and the Internet. It has been successfully applied in the fields of transportation, medical care, and agriculture. The traditional education model has defects such as low student efficiency and slow updating of educational knowledge. IoT smart education is a new type of education model, which can improve students' enthusiasm and interaction. The organic integration of artificial intelligence technology and the Internet of Things can more efficiently improve the intelligence of educational classrooms and the openness of knowledge, thereby solving the problem of unbalanced education.

The behavior information of students and teachers in remote education was selected as the research object, and it adopted the multisensor equipment of IoT, the Internet, and the terminal equipment of the computer-aided system to form the Internet of Things system. In the intelligent processing stage, the neural network method is used to extract the characteristics and time characteristics of the student behavior information and output it on the student or teacher terminal. From the information data collected by the Internet of Things, the distribution of students' speech, student behavior information, and teachers' behavior information collected by it is relatively uniform, which is conducive to the optimization process of intelligent decision-making algorithms. From the perspective of the intelligent decision-making stage of intelligent education, intelligent algorithms are more suitable for predicting student behavior information. The largest prediction error is only 2.92%, and the smallest error even reaches 0.91%. From the distribution of student behavior information, whether it is the distribution of data value or student behavior information data is consistent with the information collected by the Internet of Things.

## Figures and Tables

**Figure 1:** The workflow and equipment composition of IoT smart education.

**Figure 2:** The workflow of data fusion of IoT multisensor data source information.

**Figure 3:** The schematic diagram of the workflow of the intelligent decision-making algorithm of the IoT terminal.

**Figure 4:** The proportion of student behavior information collected by the Internet of Things system.

**Figure 5:** Differences between the student behavior information collected by the Internet of Things and the mean and minimum values.

**Figure 6:** The intelligent algorithm prediction error of intelligent education system.

**Figure 7:** The distribution of predicted value and actual value of intelligent algorithm of intelligent education.

**Figure 8:** The box distribution diagram of intelligent prediction algorithm.

**Figure 9:** The histogram of prediction algorithm of intelligent education system.

## Data Availability

The data used in this paper can be reasonably requested by readers and researchers.
